RETRACTED

# The Protective Effect of Interval Exercise on Myocardial Ischemia-Reperfusion Injury in Players

**DOI:** 10.1155/2022/4353340

**Published:** 2022-08-08

**Authors:** Wei Wang

**Affiliations:** School of Physical Education, Xi'an Physical Education University, Xi'an, 710065 Shaanxi, China

## Abstract

In recent years, the popularity of sports has been increasing. In the high-intensity competition, many players have been injured; most of them are myocardial ischemia. With the development of medical science and technology, myocardial ischemia can be reperfusion. However, sometimes, the function of tissues and organs cannot be restored, but the dysfunction and structural damage of tissues and organs can be aggravated. Therefore, it is necessary to actively carry out intermittent exercise to protect players from myocardial ischemia-reperfusion injury. The purpose of this paper is to explore the protective effect of intermittent exercise on the myocardial ischemia-reperfusion injury of players. 60 clean male Sprague Dawley (SD) old rats were selected as the research objects, which were divided into control group, ischemia/reperfusion model group, intermittent exercise + model group, and intermittent exercise + control group, and compared the parameters of heart function indexes of each group. The results showed that the creatine kinase (CK) content of control group was 0.577 ± 0.176 u/ml, lactate dehydrogenase (LDH) content was 7.834 ± 1.507 u/ml, model group was 1.257 ± 0.113 u/ml, lactate dehydrogenase (LDH) content was 14.441 ± 1.793 u/ml, intermittent exercise + model group was 0.987 ± 0.127 u/ml, lactate dehydrogenase (LDH) content was 11.714 ± 3.017 u/ml, intermittent exercise + control group was 1.103 ± 0.125 u/ml, and lactate dehydrogenase (LDH) content was 14.647 ± 2.575 u/ml. It can be seen that intermittent exercise has a good protective effect on myocardial ischemia-reperfusion injury. If the interval exercise method is integrated into the daily training of athletes, it can effectively improve the perfusion injury caused by myocardial ischemia.

## 1. Introduction

In recent years, with the process of socialization, the aging of population and the change of life style, coronary heart disease has shown a rapid growth trend among the middle-aged and old people [1]. According to the latest medical research, the incidence of coronary heart disease is about 10%, and the incidence rate is relatively high. The current clinical treatment is to restore the blood perfusion of ischemic tissue as soon as possible. The standard treatment is coronary reperfusion, including thrombolysis, percutaneous coronary intervention, and coronary artery bypass grafting [2]. In many cases, the blocked blood flow has been restored to some extent, but its tissue damage and dysfunction are further aggravated, which is clinically called myocardial ischemia-reperfusion injury [3].

RETRACTED

Exercise can also induce the expression of ischemic preconditioning (IPC) related enzymes in myocardium, such as superoxide dismutase (SOD) and constitutive nitric oxide synthase (CNOS), and exercise can induce the expression of some ischemic preconditioning related endogenous factors, such as heat shock protein 70 (HSP 70), opioid peptide, and adenosine [4]. In addition, epidemiological studies have shown that exercise can reduce the incidence and mortality of coronary heart disease, and exercise can reduce some risk factors of coronary atherosclerotic heart disease, such as effectively reduce the occurrence of diseases such as hypertension, hypercholesterolemia, and diabetes. After warm-up exercise, chest pain and ST decrease will be reduced in patients with angina [5]. Systemic and repeated exercise training before ischemia can induce myocardial ischemia tolerance, resist various secondary injury caused by myocardial ischemia, improve dysfunction, and play a protective role [6].

In recent years, many scholars have conducted in-depth research on the prevention of cardiac ischemia. Jeddi et al. found in the dog model of myocardial ischemia-reperfusion that repeated and short-term ischemic pretreatment could reduce the myocardial necrosis, arrhythmia, and myocardial systolic and diastolic dysfunction caused by subsequent ischemia/reperfusion, which provided new ideas and new approaches for the study of prevention and treatment of ischemic heart disease. It was found that high-intensity, short-term intermittent exercise can cause myocardial relative hypoxia/reoxygenation to simulate ischemia preconditioning- (IP-) induced myocardial protection [7]. Yang et al. formally put forward the concept of motion preprocessing. Exercise pretreatment means that exercise can enhance the tolerance of the heart to ischemia-reperfusion stimulation. Research shows that exercise can trigger the heart protection mechanism and produce the heart protection effect. Regular exercise can reduce arrhythmia and myocardial stunning and improve the responsiveness of coronary artery during ischemia-reperfusion, thus reducing the area of ischemia and infarction and cell death [8]. Yu et al. found that 15 minutes after the treadmill exercise test, the second treadmill exercise test was repeated again, the ischemic threshold of angina patients increased, and the myocardial oxygen consumption decreased. They believed that the increase of myocardial oxygen consumption caused by the first exercise was the main reason of warm-up exercise myocardial protection [9]. Wang et al. trained the rats on treadmill for 3 days, and ischemia-reperfusion was performed 24 hours later. It was found that exercise led to a significant increase of heat shock protein 72 (HSP 72) in the heart of rats, and the ability of the heart to resist ischemia injury was improved. It was inferred that the protective effect of exercise on the heart was related to heat shock protein 72, which also suggested that the protective effect of exercise-induced late preadaptation on the heart [10, 11].

RETRACTED

The main research content of this paper is roughly divided into four parts: the first part is the introduction part, which aims to make a systematic overview of the main research content of this paper from the research background, research purpose, research ideas, and methods; the second part is the theoretical basis, which introduces the research methods and research theories in detail and systematically. The third part is the experimental part. 60 clean male Sprague Dawley old rats were selected as the research objects, and they were divided into control group, ischemia/reperfusion model group, intermittent exercise + model group, and intermittent exercise + control group. The fourth part is the summary and suggestions of this article, which is the summary of the results of this article. The research in this paper can provide a new research direction for preventing myocardial ischemia-reperfusion injury in athletes and can also provide new ideas for the application value of interval exercise.

## 2. Proposed Method

### 2.1. Mechanism of Myocardial Ischemia-Reperfusion Injury

Myocardial ischemia refers to a pathological state in which the blood perfusion of the heart is reduced, resulting in a decrease in oxygen supply to the heart, abnormal myocardial energy metabolism, and inability to support the normal work of the heart. After ischemia for about 20 minutes, cardiomyocytes will cause immediate or gradual changes in the whole membrane system, resulting in reversible or irreversible damage [12]. The best intervention time is the first two hours, that is, the earlier effective reperfusion, the better the survival rate of myocardial cells, and the recovery of viable myocardium. Coronary artery reopening after 12 hours of ischemia can also improve the prognosis of myocardial ischemia to some extent. However, when the coronary artery is occluded for a long time, it will cause a series of irreversible damage such as necrosis of contraction band and cell lysis. For example, a major coronary artery occlusion can cause serious myocardial ischemia and apoptosis, and further cause diffuse fibrosis of myocardial tissue. It has been confirmed that fibro filaments are produced in mast cells and infiltrated fibroblasts around the ischemic area of the heart. In addition, the local vascular network and myocardial cells in the area of reperfusion showed obvious physiological and pathological changes [13, 14]. These changes can continue to aggravate myocardial tissue damage, resulting in cardiac cell dysfunction. The specific mechanisms may include autophagy, inflammatory response, energy metabolism disorders, free radical damage, calcium overload, apoptosis, and other complex dynamic changes.

RETRACTED

Neutrophils are derived from hematopoietic stem cells of bone marrow differentiation and play an important role in the nonspecific immune system when they enter the blood or tissues [15]. The cytoplasm of neutrophils contains a large number of neutral fine particles that are neither basophilic nor acidophilic and have chemotaxis, phagocytosis, and bactericidal effects. The inflammatory response caused by neutrophil infiltration is an important mechanism of myocardial ischemia/reperfusion injury, and it is also one of the reasons for the aggravation of myocardial injury and the enlargement of myocardial infarction area. The inflammatory response is activated immediately after ischemia [16, 17]. After the blood flow is restored in the ischemic area, neutrophils are introduced to the inflammatory site by chemotactic substances through adhesion, and then, a series of changes that cause myocardial cell damage occur. It mainly includes the release of no, arachidonic acid, endothelin, and prostaglandin from vascular endothelial cells, which causes vasoconstriction and blood circulation disturbance and aggravates the damage. Neutrophils have a large number of granules with enzyme activity in ischemic myocardium, among which gelatinase, collagenase, and elastase can cause serious damage to myocardial tissue [18, 19]. For example, elastase can hydrolyze important collagen, fibrin, and fibronectin in cells. The adhesion of neutrophils can make itself combine with vascular endothelial cells to change the shape. At the same time, when a large number of neutrophils are attached together, the microvasculature will be mechanically blocked, and finally, the blood circulation in the microvasculature will be blocked. During ischemia-reperfusion, neutrophils will produce a lot of free radicals. It is found that neutrophils can enhance the adhesion with vascular endothelial cells after being activated and release a lot of oxygen free radicals, which further damage the cardiomyocytes. It has been proved that exercise can improve the expression of inflammatory factors, inhibit the inflammatory response, alleviate the myocardial ischemia-reperfusion injury, and reduce the mortality and the occurrence of reinfection after myocardial infarction.

RETRACTED

In a chemical reaction, or under external influence, the covalent bond of the molecule is broken, so that the shared electron pair becomes exclusive to one side, and an ion is formed; if the result of the split causes the shared electron pair to belong to two atoms, a free radical is formed. Free radicals have strong activity and are easily affected by oxidation reaction. Therefore, oxygen radicals, including hydroxyl radicals, superoxide anions, nitrogen dioxide, and nitric oxide radicals, and lipid oxygen radicals, as well as per oxygen, singlet oxygen, and hydrogen oxide, are often encountered in biological systems, which are collectively referred to as reactive oxygen species (ROS). Under normal circumstances, endogenous oxygen free radical enzymes can clear away the active oxygen and oxygen free radicals produced in the physiological process of cell metabolism. However, when the external stimulation is too large and the self-cleaning ability is insufficient, the free radicals will be excessive and then damage the cell. When ischemia or hypoxia occurs, the balance of energy metabolism in cardiomyocytes is broken, and excessive increase of oxygen free radicals will produce lipid peroxidation reaction of cell membrane, which will cause cell damage. At the same time, a large amount of estradiol is accumulated. Once the blood supply or oxygen supply is restored, a large number of free radicals can be produced rapidly, further aggravating the ischemia-reperfusion injury. The specific mechanism of ischemia-reperfusion myocardial cell injury involves that when free radicals cause membrane lipid peroxidation, the unsaturated fatty acids of the membrane are reduced, the whole structure of the membrane is damaged, the fluidity and permeability will change, the extracellular calcium ions entering the cell will increase, which will lead to calcium overload, and the calcium overload will further accelerate the generation of free radicals, so the interaction between the two will increase the injury of bar centric muscle cells.

As an important ion of physiological activities, calcium ion can maintain the electrical balance on both sides of cell membrane and maintain the normal function of nerve conduction, nerve muscle conduction, and muscle contraction and relaxation. After the occurrence of ischemia/reperfusion, the content of calcium in myocardial cells increased significantly, and the balance of calcium was broken, which led to the phenomenon of cell injury called calcium overload. Calcium overload is one of the most important mechanisms of myocardial injury in ischemia/reperfusion. The degree of damage is positively related to the increase of calcium concentration. Therefore, calcium antagonists can effectively reduce the reperfusion injury. It mainly inhibits the influx of extracellular calcium ions by blocking calcium ion channels on the membrane of myocardial and vascular smooth muscle cells, reducing the level of intracellular calcium ions, and causing changes in the functions of cardiovascular and other tissues and organs. The occurrence of calcium overload in myocardial ischemia-reperfusion injury mainly involves the following mechanisms: the increase of cell membrane permeability, the activation of Na + ~ Ca2 + exchange mechanism, the activation of H + ~ Na + exchange mechanism, the opening of calcium channel, the decrease of calcium pump activity, and the increase of oxygen free radicals.

RETRACTED

### 2.2. Heart Protection Theory of Exercise

At present, it is believed that the cardioprotection effect of exercise pretreatment may come from two aspects: one is that exercise itself causes myocardial ischemia or relative ischemia causes myocardial relative hypoxia/oxygen enrichment to form IP mode; the other is that exercise, as a stress source, triggers some endogenous factors to cause cardioprotection effect, but the specific protective mechanism of exercise-induced resistance to I/R injury is still controversial. At present, the mechanisms proposed mainly include exercise can enhance the antioxidant capacity of myocardial tissue by upregulating ROS; exercise can improve the content of calcitonin gene-related peptide (CGRP) and affect the vasoactive; exercise can reduce the incidence of arrhythmia and cardioonia; exercise-induced heat shock protein (HSP) expression increased and myocardial contractility increased; when an organism is exposed to high temperatures, it is thermally stimulated to synthesize this protein to protect the organism itself; exercise opened sarcolemma/mitochondrial ATP-sensitive K channel (SARC/Mito KATP) to protect the heart; exercise could regulate the activity of autophagy-related proteins, improve cardiac function, and improve myocardial tolerance to ischemia and hypoxia.

The primary cause of oxidative stress in the heart is the relative or absolute lack of oxygen and oxygen in the heart. In recent years, it has been confirmed that cardiovascular stress (myocardial ischemia, ischemia/reperfusion injury, ischemic preadaptation) generally exists in exercise training. Among them, oxidative stress caused by myocardial ischemia/reperfusion and excessive exercise can cause cardiac inflammatory response, enlarged infarct area, and impaired cardiac function, but oxidative stress in ischemic preadaptation and appropriate intensity exercise can make the heart produce adaptive changes, and its mechanism is related to the protective mechanism of oxidative stress mediated by reactive oxygen species. As a direct primer for oxidative stress, endogenous reactive oxygen species (ROS) mainly exist in the form of superoxide anion, hydroxyl radical (OH), and hydrogen peroxide. ROS, as a trigger, can activate downstream Akt, mitogen-activated protein kinases (MAPK), adenosine 5′-monophosphate- (AMP-) activated protein kinase (AMPK), protein kinase C (PKC), and other protein kinases in cells, which has a positive significance in inducing cardiac signal transduction. Exercise can decrease the level of angiotensin II receptor and increase the activity of antioxidant enzymes, which has a positive effect on improving myocardial remodeling and maintaining a certain amount of ROS. The moderate increase of ROS is equivalent to the increase of mediators to improve the buffering ability of oxidative stress, facilitate gene expression and protein synthesis, and improve the adaptability of myocardium to protect the heart. Exercise can also enhance the function of ROS scavenging system and upregulate the expression of manganese superoxide dismutase (MN) SOD in mitochondrial matrix.

RETRACTED

According to the histological characteristics, electrophysiological characteristics, and functional differences of cardiomyocytes, cardiomyocytes can be roughly divided into two types, namely, working cells and autonomic cells. There is a weak inward rectifying potassium channel in cardiomyocytes, which is characterized by the channel activity being obviously inhibited with the increase of intracellular ATP concentration. It is called ATP sensitive potassium channels (KATP channels). KATP channel is a key link in the signal transduction pathway of cardiomyocytes, which is related to the myocardial protective effect induced by exercise preconditioning (EP). Under physiological conditions, the KATP channel is basically closed and does not participate in the formation of action potential when excited. But after the stimulation of metabolism, KATP channel will be activated and opened, which can cause the excitation contraction coupling of action potential and then play a role in protecting tissue cells.

Exercise, as a form of physiological stress, can cause the stress response of cardiomyocytes to activate autophagy. Appropriate intensity of exercise can maintain the stability of cells by upregulating the autophagy level and degrading the metabolic waste in cells. The adaptive change of autophagy-related protein expression can be induced by a certain intensity of exercise pretraining. The results showed that the adaptive mechanism of Beclin 1 in training might be ROS production in cells after exercise stimulation, which activated nuclear factor kappa B (NF KB) signal pathway, increased the activity of Beclin L and nuclear factor kappa B (NF KB), opened mitochondrial permeability transport channel, and increased the apoptotic factors released to cytoplasm. However, after long-term exercise and hypoxia adaptation, the decrease of ROS content in cells can effectively inhibit NF-*κ*B signaling pathway, thus reducing the apoptotic factors released to the cytoplasm, causing adaptive changes in Beclin1 and NF-*κ*B, thus reducing the damage of cardiomyocytes.

RETRACTED

## 3. Experiments

### 3.1. Experimental Preparation

1. Subjects

Clean grade SD male aged rats aged 5-18 months, weight (450 ± 20) g, clean grade feeding: temperature 21°C ± 2°C, humidity 60% ± 5%, good ventilation, free drinking water, circadian rhythm, and light 12 h/12 h alternate light and dark. The aged rats were fed in advance for 1 week to adapt to the laboratory environment before the experiment. Animal feeding and experimental operation shall strictly abide by the national regulations on the administration of experimental animals and the detailed rules for the administration and implementation. Before the test, the same batch of aged rats were screened on the running platform, and the aged rats who did not cooperate or were weak in physique could not complete the running platform training were eliminated. After careful screening, 60 clean male SD rats were obtained the aged rats were weighed and numbered, and divided into control group, ischemia/reperfusion model group, exercise pretreatment + model group, and exercise pretreatment + control group according to the random number table method. The treadmill training time is set to 5 minutes. During this time, rats that have not completed the training or do not cooperate with the training will be eliminated. After taking the corresponding intervention methods of each group, 12 rats in each group were successfully retained (*n* = 12). The basic information of subjects is shown in Table 1.

(2) Main Reagents

Protein maker: sodium dodecyl sulfate polyacrylamide gel electrophoresis (SDS-PAGE) gel preparation kit; bovine serum albumin (BSA); diaminobenzidine (DAB) chromogenic liquid; radio immunoprecipitation assay (RIPA) lysate; Tween 20; anhydrous ethanol; paraformaldehyde; 2, 3, 5-chlorinated three phenyl tetrazolium (TTC); Beclin 1 polyclonal antibody; autophagy-5 (ATG-5) polyclonal antibody; 0.9% sodium chloride injection; Bradford protein concentration test kit; trashy bromomethyl lamina methane Tris; sodium dodecyl benzene sulfonate SDS.

(3) Experimental Instrument

Dhg-9030a electric blast drying oven; super clean working table; ZH-PT animal experiment running table; Lutgendorf isolated heart perfusion experiment system; high-pressure steam sterilizer; hw1000 superconstant temperature water bath; bto1100 constant flow pump; Hattic micro 220 freezing centrifuge; - 80°C super low temperature refrigerator; wd-9405b horizontal shaking table; pl303 electronic balance.

(4) Experimental Data Processing

All data collected were analyzed by Statistical Product Service Solutions22 (spss22). The data of sample measurement are subject to normal test; those who meet the normal distribution are subject to one-way ANOVA test to analyze the differences among the four groups, expressed as mean ± standard deviation; those who do not meet the normal distribution are subject to Kruskal-Wallis test to analyze the differences among the four groups, expressed as *Q*50 (*Q*25, *Q*75) (*Q*: quartile, quartile). Chi-square test was used to analyze the differences among the four groups. The independent sample *t*-test was used to analyze the difference between groups. The paired analysis was used to measure the data of sample correlation. Firstly, the normal data was tested, and the paired group difference was analyzed by paired sample *t*-test. The paired group difference was analyzed by Wilcoxon test. There was significant difference between the above tests (*P* < 0.05 or *P* < 0.01).

RETRACTED

### 3.2. Experimental Content

Control group (CON group): to ensure the accuracy and feasibility of the experiment, after 6 weeks of free feeding, the rats were operated in vitro, and the heart was quickly connected to Lutgendorf isolated heart perfusion system, continuously and stably perfused for 180 minutes, without any special treatment before and after stopping perfusion; model group (IR group): after 6 weeks of free feeding, the rats were prepared in vitro heart Miri model, that is, the isolated heart was preperfusion balanced keeping the temperature constant at 37°C for 20 minutes, close the perfusion fluid to cause the whole heart ischemia for 40 minutes and then continue to reperfusion for 120 minutes; exercise pretreatment + model group (EP + IR group): rats after 6 weeks of exercise training, the preparation of Miri model of isolated heart in I/R group; exercise pretreatment + contrast group (EP + CON group): rats exercise training 6 weeks later, the heart was operated in vitro, and the con group was duplicated. The elderly rats in the exercise group were trained with electric running platform gradient exercise for 6 weeks, 5 days a week, starting speed of 20 m/min, time of 15 min/D, every 3 days' exercise time increased by 5 min, until the exercise time of 60 min/D, the exercise time did not change, the gradient was 0°, and the electric shock intensity was 1.0 ma.

1. Preparation of myocardial ischemia/reperfusion model in isolated perfused aged rats

Preoperative preparation: connect the perfusion system with a rubber tube, and fill the perfusion bottle with the perfusion liquid. By adjusting the height of the perfusion bottle to control the perfusion pressure of the heart, the distance between the lower end of the central tube of the perfusion bottle and the heart is generally set at 70-90 cm, which can be adjusted appropriately according to the size of the heart. The outlet of the pressure reducing valve of the 95% oxygen and 5% carbon dioxide mixed gas cylinder is connected with the filling pipe in the filling device by the filling ventilation pipe. Rotate the pressure reducing valve on the gas cylinder to make the partial pressure of the filling liquid oxygen > 600 mmHg and ventilate for more than 20 min, so as to ensure that the bubbles in the filling liquid are continuous, small, and uniform. Open the hot circulation system of the water bath, adjust the temperature to 38°C, and ensure that the temperature of the perfusion liquid in the cardiac intubation is constant at about 37°C. A little nutrient solution should be reserved in the insulated perfusion tank made of Plexiglas to maintain the temperature and humidity of the isolated heart surface. Prepare sterilized surgical instruments and oxygenated cold Krebs Hensel it (K-H) simulation solution (about 4°C). The aged rats in each group fasted 12 hours before operation, and water was forbidden 1 hour before anesthesia.

RETRACTED

Intraoperative operation: heart extraction: the aged rats were injected with pentobarbital sodium solution (50 mg/kg) for 15 minutes and then continued to be injected with heparin sodium solution (100u/100 g) for anticoagulation. After the rats were completely anesthetized, the supine position was fixed on the operating table, the skin, fat, and muscle were separated, the sternum was fully exposed, and the 2-3 intercostal aorta on the left side of the sternum was sheathed and fixed in the cardiac catheterization. Cut the root of the pulmonary artery of the heart to ensure smooth coronary perfusion. Intubation into the aorta should not be too deep, so as not to damage the aortic valve or block the coronary artery. After the heart is filled and perfused with warm K-H solution of aortic root oxygen with No.1 cotton thread, it can resume beating within limn. After 20 minutes of stable perfusion, it was determined that the beating was strong, and the rhythm was even, and the perfusion fluid could be stopped for 40 minutes of total heart ischemia. Quickly lower the chest. Gently pull the pericardium of the open heart, lift the heart with the left hand, and carefully cut the vena cava, aorta, and the surrounding tissue with the sterile ophthalmic scissors. The length of the root of the aorta is about 4-5 mm for insertion. Take out the heart quickly, and be careful not to use excessive force to prevent injury. After the heart is taken out, it is immediately placed in the prepared oxygenated 4°C K-H solution, and the residual blood inside the ventricle is discharged by gently pressing the ventricle with fingers several times to prevent the formation of clots. Perfusion of the heart: keep the perfusion liquid dropping out continuously in the cardiac intubation of the perfusion device, and control the frequency at about 60 drops/min. The whole operation process from the heart in vitro to the beginning of perfusion should be controlled within 1 min; otherwise, it is easy to cause coronary embolism or even cardiac function damage.

(2) Flag for model completion

Signs of successful ischemia: during the period of complete cardiac arrest, the surface of myocardial tissue, especially the apex of heart, gradually turns pale; the heart rate slows down, and the left ventricular development pressure and other indicators decrease; the ST segment of electrocardiogram (ECG) rises, and the T wave is high; after triphenyte-trazoliumchloride (TTC) staining, obvious white infarct area can be seen, as shown in Figure 1. Signs of successful reperfusion: the isolated heart pressure recovers about 80 mmHg within 1 min after reperfusion, and the coronary artery gets power again, that is, the heart recovers effective beating. ECG showed that ST segment decreased by more than 50%, T wave decreased, and although arrhythmia, ventricular tachycardia, ventricular fibrillation, and other conditions appeared at the beginning of reperfusion, heart rate abnormalities gradually disappeared, and heart rate gradually stabilized and maintained for several hours, suggesting the success of myocardial reperfusion model.

(3) Measurement of cardiac function indexes

The standard lead ECG was recorded by inserting needle electrode under the skin of limbs. The set point, *Q* wave, and *R* wave were observed, and the set point before ischemia, immediately after ischemia, 30 minutes after ischemia and 40 minutes after reperfusion were analyzed by BL biological function experiment system. The carotid artery was inserted into the left ventricle and connected with the baroreceptor. The arterial blood pressure, the peak systolic pressure of the left ventricle, the maximum development rate of the left ventricular pressure, and the end diastolic pressure of the left ventricle were recorded.

RETRACTED

## 4. Discussion

### 4.1. Analysis of Myocardial Ischemia-Reperfusion Injury

As shown in Table 2, the ratio of ventricular weight to body weight in the intermittent exercise training group is significantly higher than that in the quiet control group, indicating that the high-intensity intermittent exercise training can make the rat heart appear exercise-induced hypertrophy. Intermittent exercise training causes adaptive changes of cardiac morphology and structure, and sports hypertrophic myocardium appears, which is characterized by the transformation of myosin from *β* type with low activity to *α* type with high activity, capillary proliferation, reasonable ratio of capillary to muscle fiber, matching of growth of noncardiac cells with that of cardiac cells, and increased cardiac compliance.

It can be seen from Table 2 that the ratio of ventricular weight to body weight in the control group is 2.847 ± 0.191 g/kg, that in the model group is 2.147 ± 0.187 g/kg, that in the intermittent exercise pretreatment + model group is 3.265 ± 0.273 g/kg, and that in the intermittent exercise pretreatment + control group is 2.293 ± 0.126 g/kg.

Before ligation, there was no significant difference in ST segment between the groups. After ligation, the ST segment was immediately raised, twice as high as that at rest. Compared with the control group, the elevation of ST point in the model group was significantly lower at 30 minutes of ischemia and 40 minutes of reperfusion. As shown in Figure 1, the ST elevation of rats in the intermittent exercise control group was significantly lower than that in the control group at 40 minutes of perfusion, and the difference was statistically significant (*P* < 0.05).

From Figure 2, it can be concluded that the ST index of the control group is 0.108 mv when normal; the value at 30 min ischemia is 0.113 mv; the value at 40 min reperfusion is 0.122 mv. The ST index of the model group was 0.114 mv when normal, the value at 30 minutes of ischemia was 0.341 mv, and the value at 40 minutes of reperfusion was 0.324 mv. The ST index of the intermittent exercise + model group was 0.108 mv when normal; the value at 30 minutes of ischemia was 0.113 mv; and the value at 40 minutes of reperfusion was 0.122 mv. The ST index of the intermittent exercise + normal control group was 0.104 mv; the value at 30 minutes of ischemia was 0.294 ; and the value at 40 minutes of reperfusion was 0.235 mv. It is shown that intermittent exercise training has an ischemic preconditioning effect, and the mechanism may be that some endogenous protective mechanisms are initiated by exercise, such as increased expression of heat shock protein, increased expression of nitric oxide synthase, and enhanced free radical defense capacity, and cell function adjustment is precise, and so on.

RETRACTED

As shown in Figure 3, after 30 minutes of ischemia and 40 minutes of reperfusion, compared with the control group, the activities of sarcosine, lactate dehydrogenase, and aspartate aminotransferase in the model group were significantly increased (*P* < 0.01), indicating that ischemia-reperfusion caused myocardial damage. The CK and LDH activities in the intermittent training ischemic model group were significantly lower than those in the ischemic model group (*P* < 0.01); the CK and LDH activities in the serum of the intermittent exercise + model group rats were significantly lower than those in the control group (*P* < 0.01).

As can be seen from the Figure 3, the CK content in the control group was 0.577 ± 0.176 u/ml, and the LDH content was 7.834 ± 1.507 u/ml; the CK content in the model group was 1.257 ± 0.113 u/ml; the LDH content was 14.441 ± 1.793 u/ml; CK content in intermittent exercise + model group is 0.987 ± 0.127 u/ml; LDH content is 11.714 ± 3.017 u/ml; CK content in intermittent exercise + control group is 1.103 ± 0.125 u/ml; LDH content is 14.647 ± 2.575 u/ml.

### 4.2. Protective Effect of Intermittent Exercise on Myocardial Ischemia-Reperfusion Injury

As shown in Figure 4, there was no significant difference in left ventricular end diastolic pressure (LVEDP) between the groups of rats before ischemia (*P* > 0.05). After 30 minutes of ligation of the anterior descending coronary artery, the LVEDP in the control model group was significantly higher than that in the control group. The intermittent exercise control group and intermittent LVEDP in the exercise ischemia-reperfusion model group was significantly lower than that in the control ischemia-reperfusion model group, indicating that after 30 minutes of ischemia, the left ventricular diastolic function of the intermittent exercise control group, and the intermittent exercise ischemia-reperfusion model group was better than the control group; at 40 minutes of reperfusion, the interval exercise training ischemia-reperfusion model group was significantly lower than the LVEDP of the control ischemia-reperfusion model group. There was no significant difference between the intermittent exercise and the control ischemia-reperfusion model group, indicating that the interval after reperfusion was intermittent. The diastolic function of the left ventricle in the exercise training group was partially restored.

RETRACTED

LVEDP represents the left ventricular preload, which reflects the diastolic function and compliance of the left ventricle. From the analysis of the above data, it can be seen that after acute myocardial ischemia and reperfusion, the left ventricle's systolic and diastolic functions are reduced, but intermittent exercise training has a protective effect on the myocardial systolic and diastolic functions. When myocardial ischemia-reperfusion injury occurs, from the perspective of cardiac function, the resting tension gradually increases with the prolongation of ischemic time, and the development tension gradually decreases. During reperfusion, the resting tension increases further, and the development tension further decreases, indicating that the myocardial contractility decreases.

As shown in Figure 5, the area of myocardial infarction in the model group was 24.4% ± 2.3%, and the area of myocardial infarction in the exercise + model group was 12.1% ± 1.7%. Compared with the model group, the area of myocardial infarction in the exercise + model group was reduced, and the difference was statistically significant (*P* < 0.05); there was no significant change in the area of the control and exercise + control myocardial infarction.

The experimental results showed that after 180 minutes of balanced heart perfusion in vitro, the myocardial infarction area of the control group and intermittent exercise + control group remained almost unchanged. A significant range of myocardial infarction appeared in the heart of the model group rats; the myocardial infarction area accounted for 24%, indicating that myocardial ischemia/reperfusion injury can cause obvious myocardial infarction. The morphological perspective proved the success of the myocardial ischemia-reperfusion injury (MIRI) model in this experiment. Compared with the model group, the area of myocardial infarction in the aged rats of the intermittent exercise + model group was significantly reduced, suggesting that exercise preconditioning can induce myocardial ischemic tolerance, inhibit apoptosis, reduce the area of myocardial infarction, and resist myocardial ischemia in old rats reperfusion injury.

## 5. Conclusions

1. The research background of this paper is that in recent years, the popularity of this is increasing. In the high-intensity competition, many players have been injured; most of them are myocardial ischemia. With the development of medical science and technology, myocardial ischemia can be re perfusion. However, sometimes, the function of tissues and organs cannot be restored, but the dysfunction and structural damage of tissues and organs can be aggravated. Therefore, it is necessary to actively carry out intermittent exercise to protect players from myocardial ischemia-reperfusion injury
2. The purpose of this paper is to explore the protective effect of intermittent exercise on the myocardial ischemia-reperfusion injury of players. 60 clean male SD old rats were selected as the research objects, and they were divided into control group, ischemia-reperfusion model group, intermittent exercise + model group, and intermittent exercise + control group. The old rats in the exercise group were trained with electric running platform gradient exercise for a period of time 6 weeks, 5 days a week, the initial speed is 20 m/min, the time is 15 min/D, every 3 days' exercise time increases 5 min, until the exercise time is 60 min/D, the exercise time does not change, the slope is 0°, and the electric shock intensity is 1.0 Ma. Finally, the heart function parameters of each group were compared
3. The experimental data showed that the set index of the control group was 0.108 mv in normal condition, 0.113 mv in 30 minutes of ischemia, and 0.122 mv in 40 minutes of reperfusion. The set index of the model group was 0.114 MV in normal condition, 0.341 MV in 30 minutes of ischemia and 0.324 MV in 40 minutes of reperfusion. In the intermittent exercise + model group, the set index was 0.108 mv in normal, 0.113 mv in 30 minutes of ischemia, and 0.122 mv in 40 minutes of reperfusion. The set index of the intermittent exercise + control group was 0.104 mv in normal condition, 0.294 mv in 30 minutes of ischemia and 0.235 mv in 40 minutes of reperfusion. In this paper, the protective damage of myocardial ischemia-reperfusion has been deeply studied, but due to the limited experimental conditions, there are still many shortcomings in this paper, and the research quality will be continuously improved in the future work

RETRACTED

## Figures and Tables

**Figure 1:** Myocardial ischemia pathological images.

**Figure 2:** ST changes in each group.

**Figure 3:** Serum myocardial enzyme levels in each group.

**Figure 4:** Comparison of LVEDP values.

**Figure 5:** Myocardial infarction area ratio.

**Table 1:** Basic information of subjects.

	Age	Temperature	Weight
Con group	9	21 ± 2	460.7 ± 12.80
Ischemia/reperfusion group (I/R group)	10	21 ± 2	451.45 ± 16.40
Exercise preprocessing+ischemia reperfusion group (EP + IR group) Exercise preprocessing+control group (EP + CON group)	11 10	21 ± 2 21 ± 2	458.09 ± 14.39 448.68 ± 14.56

**Table 2:** Changes of the ratio of ventricular weight to body weight.

Group	Con group	IR group	EP + IR group	EP + CON group
Ventricular weight/weight	2.847 ± 0.191	2.147 ± 0.187	3.265 ± 0.273	2.293 ± 0.126

## Data Availability

No data were used to support this study.
